# Risk Assessment of Hip Fracture Based on Machine Learning

**DOI:** 10.1155/2020/8880786

**Published:** 2020-12-22

**Authors:** Alessio Galassi, José D. Martín-Guerrero, Eduardo Villamor, Carlos Monserrat, María José Rupérez

**Affiliations:** ^1^Intelligent Data Analysis Laboratory (IDAL), Dept. of Electronic Engineering, ETSE-UV, Universitat de València, Avinguda de la Universitat s/n. 46100 Burjassot, València, Spain; ^2^Centro de Investigación en Ingeniería Mecánica (CIIM), Universitat Politècnica de València, Camino de Vera s/n, 46022 València, Spain; ^3^VRAIN, Universitat Politècnica de València, Camino de Vera s/n, 46022 València, Spain

## Abstract

Identifying patients with high risk of hip fracture is a great challenge in osteoporosis clinical assessment. Bone Mineral Density (BMD) measured by Dual-Energy X-Ray Absorptiometry (DXA) is the current gold standard in osteoporosis clinical assessment. However, its classification accuracy is only around 65%. In order to improve this accuracy, this paper proposes the use of Machine Learning (ML) models trained with data from a biomechanical model that simulates a sideways-fall. Machine Learning (ML) models are models able to learn and to make predictions from data. During a training process, ML models learn a function that maps inputs and outputs without previous knowledge of the problem. The main advantage of ML models is that once the mapping function is constructed, they can make predictions for complex biomechanical behaviours in real time. However, despite the increasing popularity of Machine Learning (ML) models and their wide application to many fields of medicine, their use as hip fracture predictors is still limited. This paper proposes the use of ML models to assess and predict hip fracture risk. Clinical, geometric, and biomechanical variables from the finite element simulation of a side fall are used as independent variables to train the models. Among the different tested models, Random Forest stands out, showing its capability to outperform BMD-DXA, achieving an accuracy over 87%, with specificity over 92% and sensitivity over 83%.

## 1. Introduction

The continuous increase in life expectancy also raises the incidence of problems related to the weakening of the body due to age. Among the diseases and medical conditions that afflict the countries of the first world, next to the cardiovascular and nervous system ones, but very underestimated in comparison, there are the problems related to bones. In particular, one of the biggest problems for people over 65 is hip fracture due to osteoporosis. Osteoporosis is a skeletal disease primarily characterized by reduced bone mass [1].

According to data from the International Osteoporosis Foundation (IOF), approximately 1.6 million hip fractures occur around the world each year, and in 2050, this number will increase to figures between 4.5 and 6.3 million, due mainly to the aging population [2]. In addition, it is also estimated that about 75% of all fractures occur in women, due to the accumulation of certain risk factors that are linked to gender. In the case of Spain, in 2015, this disease was suffered by 2.2 million women and 0.6 million men, which is practically 1% of the current Spanish population. According to the IOF, it is also estimated that around 330,000 fragility fractures occurred in this country in 2017.

The gold standard for osteoporosis diagnosis and hip fracture risk assessment is currently the Bone Mineral Density (BMD), which is measured by Dual-Energy X-Ray Absorptiometry (DXA) [3]. However, its ability for discrimination between fractured and control cases is limited. BMD distributions for aged people of both groups overlap to a large extent, reducing the classification accuracy to about 65% [4]. Alternative methods have been proposed to calculate the risk of fracture as FRAX and the Garvan [5, 6]; they are statistical models based on clinical variables in which patient data are compared to a large database from the USA population that includes many clinical features: age, gender, previous fractures, etc. The classification accuracy is about 70% [7], which is not a significant improvement compared to BMD. Another alternative method is measuring the volumetric distribution of the BMD (vBMD) by quantitative computed tomography QCT, which is considered to be more sensitive for osteoporosis [8]. However, although QCT allows to obtain the three-dimensional geometry of the bone and provides the volumetric distribution of BMD, QCT is not integrated in the clinical routine because of its higher cost, processing time, and radiation exposure [9].

Other radically different approaches are the data-based strategies, which consist in training a Machine Learning (ML) model from simulations (e.g., obtained from finite element methods (FEM)) or directly from clinical data. ML algorithms are able to automatically learn nonlinear mappings between several inputs (clinical data, biomechanical data, etc.) and several outputs (e.g., fracture risk factors). Although the training process is relatively slow, once trained, these algorithms provide extremely quick inference times, therefore fulfilling the requirement to predict solutions in real time [10]. This situation opens a possibility to use FEM to generate data off-line that ML models can use to estimate a function that maps inputs (mechanical properties, geometry mesh, boundary conditions, etc.) and outputs (nodal displacements, stresses, strains, etc.) [11] to provide valuable fracture risk predictors in real time.

Machine Learning (ML) has become a robust and relatively usual approach to use in dealing with complex data in order to extract unexpected risk factors in the field of preventive medicine [12]. However, the literature only shows a few studies related to the assessment of the osteoporosis hip fracture. One of the mentioned works can be found in [13]. In this work, a clustering analysis for identifying subgroups of osteoporosis Danish patients based on similarities of traits was carried out. Nine patient clusters of different fracture risks were identified making use of a dataset made up of 10,775 subjects. Four clusters represented postmenopausal women with high-fracture risk profiles of low BMD and between-group differences of poor versus good antiresorptive treatment compliance. One cluster formed by 9% of the subjects was particularly worrisome due to the poor treatment compliance and the very low BMD. Three clusters representing the majority were women with average-fracture risk profiles. Finally, two clusters of perimenopausal and very young women represented low-fracture risk subjects with high BMD and low comorbidity. The authors claimed that for patients older than 60 years a clear distinction between groups of high-fracture risk and average-fracture risk was achieved.

Another remarkable work can be found in [14], where artificial neural networks (ANN) were used to predict hip fracture. The data included information about age, BMD, clinical factors, and lifestyle factors which had been obtained from a longitudinal study that involved 1167 women aged 60 years and above from Dubbo, Australia. The women were followed up for up to 10 years, and during the period, the incidence of new hip fractures was ascertained, although only 90 sustained a hip fracture. Two models were developed: the former was produced by combining only lumbar spine and femoral neck BMD and the latter non-BMD factors, with accuracies of 82% and 84%, respectively. A third model was produced by combining BMD and non-BMD factors, reaching an accuracy of 87%. In summary, the authors showed that ANNs were able to predict hip fracture more accurately than other existing statistical models. However, in spite of the good results, no mechanical attributes were included into the models; as they are considered the main responsible factors for bone failure, this might limit the accuracy of the model if applied to a different dataset.

The mechanical behaviour of the femur during a sideways fall is the main responsibility of hip fracture. In fact, the comparison of the impact load at the fall with the femur strength will determine the bone failure. It is true that BMD is the main contributor to the femur strength, but most of the statistical models do not carry out this comparison to predict hip fracture. Obtaining the mechanical characteristics of the bone has been commonly addressed in the literature by finite element (FE) approaches. QCT-based models construct a biomechanical model from the 3D geometry of the bone and the 3D volumetric distribution of the BMD, which is used to obtain the material properties of the bone [15, 16]. However, even though they are pretty accurate models, its hard implementation, limitations, and computational cost make them unfeasible to be used in clinical routine. In contrast, FE models based on DXA construct the biomechanical model from a 2D representation of the bone and a 2D distribution of the BMD. Therefore, its implementation is easier and their computational cost is lower. In addition, they are very attractive for clinical practice since they do not interrupt the current clinical workflow. These models have provided estimates of the bone strength and have increased the classification accuracy to about 80% [17–19]. Furthermore, fracture risk and Hip Structural Analyses (HSA) derived from both QCT and DXA-based models seem to be significantly correlated [20].

There are some studies that have used ML techniques combining both clinical data and mechanical data. Nishiyama et al. [21] performed patient-specific QCT-based FE analyses under multiple loading conditions to feed a Support Vector Machine (SVM) classifier with a radial basis kernel to address uncertainty in the fall configuration. Jiang et al. [22] investigated the combination of clinical and FE-derived mechanical attributes by means of SVM using a fully parameterized three-dimensional FE model that was created using the given values of geometric attributes; however, this model was global instead of patient-specific. A recent study used high-resolution Magnetic Resonance Imaging- (MRI-) derived data to compare 15 ML classifiers at predicting any kind of osteoporotic fracture [23]; the data comprised bone tissue elasticity and topology of the proximal femur at specific volumes of interest computed with microfinite elements; although this study gave some insight into the relevance of microstructural parameters, the dataset was small and it was not specially focused on hip fracture. It is important to notice that in all these studies the authors did not use a FE model including patient-specific data describing geometry or BMD distribution. Our conjecture is that including mechanical attributes into a ML model may enhance hip fracture prediction rather than using clinical attributes alone.

In the field of osteoporosis and hip fracture risk assessment, supervised Machine Learning has been scarcely applied in conjunction with computationally driven mechanical attributes. Our group recently published a study where supervised Machine Learning was applied in conjunction with clinical and computationally driven mechanical attributes [24]. A total number of 137 postmenopausal women aged 81.4 ± 6.95 were included in the study and separated into a fracture group (*n* = 89) and a control group (*n* = 48). A semiautomatic and patient-specific DXA-based FE model was used to generate mechanical attributes describing the geometry, impact force, bone structure, and mechanical response of the bone after a sideways fall. After preprocessing the whole dataset, 19 attributes were selected as predictors. SVM with radial basis function (RBF), Logistic Regression (LR), Shallow Neural Networks, and Random Forests (RF) were tested through a comprehensive validation procedure to compare their predictive performance. The results showed that SVM generated the best-learned algorithm for both experimental setups, when clinical and mechanical attributes were included and also when only clinical attributes were taken into account. The first setup generated the best-learned model outperforming the accuracy of BMD by 14pp (79%).

This paper enhances the study presented in [24] by making use of clinical, geometric, and biomechanical variables of the previous database followed by a relevance ranking to find out which variables are the most important ones for the problem. With the selected variables, different ML models were trained. The results show that RF is the best option with an accuracy over 87%, specificity over 92%, and sensitivity over 83%. These values are much better than the current BMD clinically used whose classification accuracy is around 65% and also better than the accuracy of our previous work that was 79%. On top of that, the use of data generation techniques is also remarkable to balance the number of samples in the two classes that were biased originally.

The rest of the paper is outlined as follows.  Section 2 presents the methods as well as the characteristics of the dataset and the process to select attributes. The achieved results are shown in Section 3, ending up the paper with the concluding remarks and our proposals for the future research in Section 5.

## 2. Material and Methods

### 2.1. Biomechanical Model

#### 2.1.1. Study Population

The database was the same used in [24]. A total number of 137 patients were included in the study with a mean age of 81.4 ± 6.95 years. The inclusion criteria comprised postmenopausal women, older than 50 years, with clinical risk factors related to osteoporosis. Women showing evidence of hip fracture were recruited after being admitted to the emergency room of Hospital Mútua Terrassa (Terrassa, Spain). A densitometry exploration was indicated for each subject.

The scans were performed at CETIR Medical Group, after informed consent was obtained. The time between fracture and DXA acquisition was less than two weeks. DXA scans were taken on the opposite femur to the fractured one using GE Healthcare Prodigy Advance bone densitometer (GE Healthcare, Madison, WI, USA). Subjects were placed on the DXA table in the prone position, with feet parallel to the table and a leg internal rotation of 25-30°, according to the manufacturer's recommendations. The image pixel size was 0.6 mm × 1.05 mm. Patients were separated into a fracture group (*n* = 89), with fall-related incident hip fracture, and a control group (*n* = 48). Within the fracture group, 45 accounted for a trochanteric fracture and 44 for a neck fracture.

#### 2.1.2. Patient-Specific FE Model

A 2D patient-specific FE model was created aimed at obtaining the mechanical attributes to be used in the ML models [24]. For each DXA scan, the proximal femur was segmented manually (Figure 1). Regions of interests (ROIs) defining the trochanteric and neck region were defined semiautomatically. The inputs required for the construction of the FE model were the segmented image of the femur, along with the basic clinical information of the patient (height, weight, and gender).

After the segmentation, the process does not require human interaction. The femur shaft is rotated 10 degrees to the physiological configuration. Pads are placed covering the femoral head and the greater trochanter to avoid local damage due to the applied boundary conditions [25, 26]. The femur, trochanteric pad, and femoral head pad are meshed using TetGen [27]; following a convergence analysis, the mesh size was defined with approximately 60,000 elements, depending on the subject. The model was built under the assumptions of plane strain and linear elasticity behaviour.

The bone material properties were calculated from the BMD per pixel, using the empirical equations obtained in [28–30]. The Poisson ratio was set to 0.3 [31]. Based on previous studies involving mechanical tests [32] and FE models [33], the PMMA (Polymethylmethacrylate) material properties, 1.5 GPa for the Young modulus and 0.37 for the Poisson's ratio, were used for the pads. The heterogeneous material distribution obtained for the Young's modulus is shown in Figure 2(a). This figure shows how the elastic modulus varies according to the BMD distribution from the femur shown in Figure 1.

To obtain the mechanical attributes, a sideway fall was simulated with the FE patient-specific model for each patient. The open-source FE package FEBio [34] was used to obtain the numerical solution. Regarding the boundary conditions, the displacement of the nodes at the distal end of the femoral shaft was totally restricted, and the medial displacement of the nodes at the femoral head pad was prevented.  Figure 2(b) specifies the location of the applied loads as well as the location of the boundary conditions. The load was applied to the greater trochanter through its pad, representing the fall-related impact force [35, 36]. This load was calculated with the mass-spring impact model of [37], whose input variables were the weight, the height, and the gender of the patient. Once the peak impact force (FPK) was obtained, the attenuated impact force (FP) was calculated subtracting the attenuation force: FAT = 71 · STH, based on previous studies regarding the effect of soft tissue thickness (STH) [38] and correlations between body mass index (BMI) and STH [39]. Finally, the applied load pressure over the hip (HP) was computed dividing the attenuated impact force by the length of the greater trochanter pad (*b*) and a subject-specific thickness (*t*) [24].

### 2.2. ML Models

#### 2.2.1. Inputs to the ML Models

Five groups of attributes where collected for each patient [24]: clinical, geometrical, fall-related, bone tissue-related, and that derived from the FE analysis (FEA).  Table 1 shows the clinical attributes obtained from the clinical report; mean values and standard deviations (SD) are provided for each attribute and both groups (fractured and control).

The general scheme to obtain the geometrical attributes is shown in Figure 3. This figure graphically describes the geometrical attributes to introduce in the model. These attributes were obtained through a morphometric analysis performed on the proximal femur geometry [19]. Their values are shown in Table 2.

The fall-related attributes computed for each patient are shown in Table 3. Regarding to bone tissue structural properties, the cortical bone was defined as having an apparent density greater than 1.0 g/cm^3^ [33]. The percentage of the trabecular bone (TB) and cortical bone (CT) within the femur bone was estimated using this threshold as well as the average Young's modulus within each tissue (TBE and CTE). These values are shown in Table 4.

From the FE linear simulation of the side-fall performed with FEBio, several mechanical attributes were selected and they are shown in Table 5; some of them were computed to define the failure of the whole bone as the load-to-strength-ratio (LSR) and the femoral strength (FS), following the criterium of [15]. LSR was defined as the minimum ratio in a contiguous area of 9 mm^2^. This area comprised the elements with the highest ratios between the Principal Compressive Strain and the Compressive Yield Strain. The most common sites for femur fracture are the neck and the trochanteric regions. Because of this, mechanical attributes at each region were computed (index *N* is used for the variables at neck region, and index *T* for the variables at the trochanteric region). The volume weighted average value of maximum and minimum principal stresses (*S*_1_ and *S*_3_), the maximum and minimum principal strains (*E*_1_ and *E*_3_), the major principal stress (MPStress), the major principal strain (MPStrain), the strain energy density (SED), and the fracture risk index (FRI) were computed. MPStress and MPStrain were defined as the maximum eigenvalue in the stress and strain tensor, respectively. FRI was computed as the weighted average ratio between the Von Mises stress and the yield stress in the region.

To build the model, the cohort (137 patients) was divided into training (70% of the data) and test (the remainder 30%) with an equal distribution of fractured and healthy patients. Since the number of subjects used for training might be insufficient to obtain conclusive results, Synthetic Minority Over-sampling Technique (SMOTE) was used [40]. The goal of using SMOTE is two-fold: the first one is to increase the size of the dataset so that models can be trained with a more meaningful information and have more parameters without overfitting the data, and the second one is to balance both classes (fractured and control). Classification models may worsen their performance when dealing with unbalanced classes; hence, by creating synthetic samples, both classes can have a similar number of samples. In particular, the number of samples was increased up to 400 distributed in 200 of healthy and 200 of fractured samples. For the sake of reliability, the synthetic samples produced by SMOTE were only applied to the training set in order to ensure that potentially incorrect synthetic points did not affect the models eventually obtained.

#### 2.2.2. Attribute Selection Process

After a process of attribute normalisation, the selection of the most significant attributes was performed in two steps: Principal Component Analysis (PCA) and correlation analysis.  Table 6 shows the percentage of variance included in the 39 components of the PCA. Thus, the first principal component (with the 91.88% of the accumulated variance) is clearly dominant compared to the rest. Moreover, adding the second and the third components, we can represent 99% of the total variance of the dataset. Since PCA is a linear combination of all the attributes, it is necessary to analyse the contribution of each one to the linear combination. As most of the attributes have very low weights (between 10^−3^ and 10^−15^), their contribution can be deprecated. Those principal attributes with significant contribution (weights ≈1) to the first six principal components are the following:

- PC1: TB and CT
- PC2, PC3, and PC4: BMI, STH, FPK, FAT, and FP
- PC5: BMD, HP, FRI_N, and FRI_T
- PC6: BMD, HP, TBE, LSR, FRI_N, and FRI_T

Focusing on the three first principal components that, as mentioned above, contain 99% of the variance, only seven make a contribution:

- TB: ratio of trabecular bone
- CT: ratio of cortical bone
- BMI: body mass index
- STH: soft tissue thickness
- FPK: peak impact force
- FAT: force of attenuation
- FP: attenuated impact force

Additionally, to the PCA Analysis, a correlation analysis was performed: Pearson's correlation index and Spearman's Rank correlation index were obtained.  Figure 4 shows Pearson's correlation index of all 39 attributes. The coloured squares with ones inside mark the pair of attributes with correlation higher than 0.9; all except one of the high-correlated attributes were hence removed in order to reduce the dimensionality of the problem.

Pearson's correlation is based on two hypotheses: the populations are normally distributed and the subpopulations do not have the same variance. If at least one of the two hypotheses fails, Pearson's index should not be applied. To avoid these limitations, we have also made use of Spearman's correlation that basically translates the values into ranges before calculating the correlation coefficients. As in the previous case, Figure 5 shows the corresponding heat map.  Figure 6 joins Spearman's and Pearson's correlations in a single visualisation.Starting from the seven variables selected by the PCA, our proposal is to include some additional features as the result of the correlation analysis. In particular, we considered those variables which correlated with (at least) four other attributes not previously included by the PCA. The columns of Table 7 show the most highly-correlated variables not previously included by the PCA and the rows those features linked to them with a correlation higher than 0.9 (marked with the check sign). These are HP, S3_N, FRI_N, and FRI_T. It is remarkable that only four features can include most of the information stored in 18 variables.

A final analysis was done for those features already selected by the PCA but with a high interdependence according to the corresponding correlation coefficients, namely, BMI, FAT, and STH. In particular, FAT is calculated as follows:

(1) $$\begin{array}{c} \text{FAT}=71\times \text{STH}\left(\text{g}/{\text{cm}}^{2}\right), \end{array}$$

while STH is (for female patients) as follows:

(2) $$\begin{array}{c} \text{STH}=2.3451\cdot \text{BMI}-33.4440\left(\text{g}/{\text{cm}}^{2}\right), \end{array}$$

And hence,

(3) $$\begin{array}{c} \text{FAT}=71\cdot \left(2.3451\cdot \text{BMI}-33.4440\right)\left(\text{g}/{\text{cm}}^{2}\right). \end{array}$$

Due to this high interdependence, FAT and STH were removed because BMI is more easily and routinely collected. Besides, it can also be observed that TB and CT are linked by a strong correlation. In fact,

(4) $$\begin{array}{c} \text{CT}+\text{TB}=1. \end{array}$$

Therefore, only one attribute is enough to include the information provided by the two. The variable TB was eventually selected. Summing up, eight attributes out of 39 were finally used to build the ML models. These eight attributes actually included information related to 26 out of the 39 attributes according to the correlation analysis (Table 8).

#### 2.2.3. Fracture Discrimination

To build the classifier, we considered some of the most popular ML approaches: LR, SVM, Decision Trees (DT) and RF. All the models were trained considering that the positive class—coded as 1—corresponds with fractured patients and the negative class—coded as 0—with control samples. The goodness of the models was assessed by means of sensitivity (Se), specificity (Sp), and accuracy (Acc).

LR was obtained after 1000 trials, randomly selecting the training and test sets. After this random selection, SMOTE was applied to the training set to increase the number of training samples. We also analysed if increasing the number of predictive attributes could improve the prediction results. The features that were added for this analysis were NW, NSA, FA, and SAL that were the lowest correlated attributes not previously considered. A clear degradation of the results was observed when including even more attributes.

As the data set is considerably sparse, SVM could be a good option to model it. Different kernels were considered: linear; linear with posterior probability regions; sigmoid; sigmoid with posterior probability regions; Gaussian; Gaussian with posterior probability regions; and Bayesian with posterior probability regions. As in the case of LR, each SVM was run 1000 times with random selection of training and test sets.

With respect to DT, the same experimental setup was taken into account. The Gini score was used as a splitting criterion. Finally, RF also followed the same training procedure. Different architectures were considered trying to avoid overfitting by limiting the number of trees and their depth.

## 3. Results

The mean values, standard deviations, and best result among the 1,000 runs are shown in the tables describing the performance of the different models; all results correspond with the test sets. The eight attributes selected as the result of applying PCA and correlation were taken into account; besides, an analysis with 12 features adding the four features mentioned in Section 2.2.3 was also considered.

### 3.1. Logistic Regression

Tables 9 and 10 show the results achieved by LR using eight and 12 predictive attributes, respectively. Although the best model does yield a very powerful result, the mean values of Se, Sp, and Acc slightly improve the ones provided by the widely used BMD. There are no meaningful differences between the results obtained with eight or 12 features.

### 3.2. SVM Models

The results obtained by the seven SVM models described in Section 2.2.3 are shown in Tables 11–17. There is a remarkable difference between Se and Sp. Obviously, a model capable of classifying well both classes is always desired, but if the model has to be biased to one of the classes and in order to have a model useful for its real application, sensitive models are preferred. As a result, the number of false negatives is very low, and hence, the predictive capability to detect fractured patients is very high. This is why in order to achieve an Acc as high as possible, we decided to bias the model towards Se. The obtained models are sensitive enough, but unfortunately, the Sp is so poor (near 50%) that would not justify its actual use as a clinical decision support system (CDSS). SVM in general do not benefit from the inclusion of the four additional features.

### 3.3. Decision Trees

Table 18 shows the results achieved by DT. They do not benefit from the use of the additional features, likely because it reduces the density of branches in the tree and hence its ability to find homogeneous groups of patients. The results are slightly worse than those provided by LR and quite close to what BMD can attain. The standard deviations are too large suggesting the low reliability of the modelling.

### 3.4. Random Forest

In the case of RF, the robustness of the model is in its own design formed by many single DT so the experimental setup of 1,000 runs was not considered here. For the sake of a fair comparison, RF were made up of 1,000 trees. Therefore, no mean values and standard deviations are given in Table 19, which describes the RF results. The inclusion of the four additional features has a positive effect in the RF performance, slightly improving Se, Sp, and Acc. RF provides the best results of all the tested models with great prediction capabilities for both classes, turning out to get an Acc of 87%, well above the Acc reported by BMD.

Although this work can be considered a pilot study, the promising results yielded by RF encourage us to carry on with the study, hopefully increasing the size of the dataset. If RF performance is similar when applied to a large cohort of subjects, we reckon that its use as CDSS should be taken into account.

## 4. Discussion

As has been shown, the Linear Regression approximation has quite poor results. The low ratios of sensitivity, specificity, and accuracy only a little over 70% with extremely high standard deviation (higher than ±10%) transform Logistic Regression in a bad approximation. Bearing in mind, in addition, there can be no underfitting (we got 200 samples because of the use of SMOTE) and neither overfitting, as 8-12 features are less than a tenth of the number of subjects. It can be observed that using more attributes does not significantly improve the behaviour of the model.

With regard to the SVM, it is clear that the sigmoid totally misunderstands the “shape” of the hyperplane. The highest value given is 61% of specificity, for 12 features. Accuracy does not move from values around 57-58% that is quite lower that actual models based only on BMD that achieves an accuracy around 65% (see Section 1). Linear kernel returns sensibly higher results, but nothing considerable good: while specificity increases around 75-77%, the sensitivity is still lower than 70%. Following, the maximum accuracy is lower than 72%.

Bayesian kernel, along with PPR, increases a little bit the numbers: considering 12 features, the sensitivity is around 71%, the specificity is 10% higher, and the accuracy overreaches the 75%. Finally, using a Gaussian kernel, the sensitivity builds on a lot, reaching values up to 83% (8 features) and for the simple elaboration, and almost 94% for the Gaussian + PPR, handling 12 features. Both with and without PPR, the accuracy overreached 80% of accuracy.This is the best result obtained for the SVM modeling and reaches levels of the state of the art published to date (see Section 1).

On the other hand, Decision Trees do not return good results. Generally, the values for sensitivity, specificity, and accuracy are lower than SVM (considering the best fitting kernels). On the other hand, the standard deviation is sensibly greater (in average) than all the previous models, being the weak spot of this model. Accuracy is good, but sensitivity and specificity are unbalanced, in favor of the latter. For both 8 and 12 predictive attributes selected, the accuracy is around 65-66%.

Finally, Random Forest is the best among all the built models. Although the model built with only 8 features is less precise (around 5% for each value) than the one built with 12, it outrages the results obtained by models published until now. We have also observed that adding more attributes (up to 15), the results do not improve significantly, so the best move is to keep 12 features to grant a lighter dataset. In conclusion, neither of the previous models obtain such great results: 83% for sensitivity, 92% for specificity, and an accuracy of 87%.

As it was commented in Section 1, this paper enhances the study presented in [24]. The same clinical, geometric, and biomechanical variables of the previous database were used in this paper. However, this paper presents some novelties that improve our previous work. One of them is the relevance ranking carrying out to find out which variables are the most important ones for the problem. In our previous work, this ranking was performed only studying Pearson's correlation. In the present work, the relevance ranking was performed in two steps: Principal Component Analysis (PCA) and correlation analysis, analyzing both Pearson's correlation index and Spearman's Rank correlation. However, the true improvement was obtained by the Principal Component Analysis.

As PCA is based on a reduction of the problem dimensions keeping the maximum information, our models are more precise, with more capability of generalization to be applied to new data and with more capability of interpretation for the post-processing of the results.

Another improvement is related to the application of the SMOTE technique in order to increase the number of training samples, which improved the results of our models. Finally, ML models different to those used in our previous work were used in this work as Decision Trees (DT) and Random Forest (RF), which provided with better results in terms of sensitivity, specificity, and accuracy. In fact, RF was the best option with an accuracy over 87%, specificity over 92%, and sensitivity over 83%. These values are much better than the current BMD clinically used whose classification accuracy is around 65% and also better than the accuracy of our previous work that was of 79%.

One of the main limitations of the present study was the sample size. Although the sample size was larger than other studies, it is still not larger enough, which might limit the learning process. Another of the limitation of this study is related to the resolution of the images. Pixel size was approximately 8 times greater than in other commercial densitometers (e.g., GE Healthcare iDXA Advance), thus providing low resolution images. The discriminative power of FEM-derived attributes highly depends on the material properties, which are extracted from the BMD maps. The details of these maps depend on the quality of the image, and if the image resolution is low, some information might have been lost.

There exits an inherent limitation in the present study due to the 2D model, which is developed on the overlapping of cortical and trabecular bone on the image plane. Therefore, stress and strain distributions may be altered, and the failure starting location might not be fully reliable. On the other hand, as it was commented previously, we could not construct ML models that differentiate between neck and trochanteric fractures due to the size of the dataset. Finally, although our study focused on prediction of hip fracture in postmenopausal women, hip fracture also happens in the male population [41]. Moreover, differences between male and female fracture attributes, both clinic and biomechanical, have been shown in the literature. This should be addressed in order to build an effective predictive model for both genders.

## 5. Conclusions

This paper proposes the use of Machine Learning (ML) models trained with data from a biomechanical model that simulates a sideway fall, aimed at improving the accuracy of the current gold-standard in osteoporosis clinical assessment. The current gold standard is Bone Mineral Density (BMD) measured by Dual-Energy X-Ray Absorptiometry (DXA), and its classification accuracy is only around 65%. Among the different tested models, Random Forest stands out, showing its capability to outperform BMD-DXA, achieving an accuracy over 87%, with specificity over 92% and sensitivity over 83%.

This paper enhances the study presented in [24]. The same clinical, geometric, and biomechanical variables of the previous database were also used in this work. However, this paper presents some novelties that improve it, as the relevance ranking carried out to find out the most important ones for the problem, which was performed by PCA. Thus, the models developed in this work were more precise, with more capability of generalization to be applied to new data and with more capability of interpretation for the postprocessing of the results.

The application of the SMOTE technique to increase the number of training samples also improved the models. In addition, different ML models to those used in our previous work were used in this work: Decision Trees (DT) and Random Forest (RF), which provided with better results in terms of sensitivity, specificity, and accuracy. These values were much better than the current BMD clinically used whose classification accuracy is around 65% and also better than the accuracy of our previous work that was of 79%.In conclusion, this study has shown that hip fracture prediction can be modelled by a multitechnique approach, considering clinical and biomechanical data into a ML classifier. This approach is economical and fast and could be integrated in the clinical routine without changing the clinical workflow. Future research works should include a greater 480 volume of samples, better image quality, and more specific predictions of the fracture location.

## Figures and Tables

**Figure 1:** Original image from the iDXA densitometer database enhanced by a Gaussian filter (a). Manually segmented image (b).

**Figure 2:** Material properties, loading, and boundary conditions automatically generated.

**Figure 3:** Graphical description of geometrical attributes [24].

**Figure 4:** Pearson's correlation: heat map considering a threshold of 0.9. The white zeros represent a correlation lower than the threshold while the coloured ones stand for a correlation equal or higher than 0.9.

**Figure 5:** Spearman's correlation: heat map considering a threshold of 0.9.

**Figure 6:** Heat map result of joining the information provided by Person's and Spearman's indices: the black squares represent a correlation higher than 0.9 while the white zeros indicate that the threshold is not reached.

**Table 1:** Clinical attributes.

	Clinical attributes		
Attribute	Description	Fractured (mean ± SD)	Control (mean ± SD)
Age (years)	Patient's age	81.39 ± 6.98	82.56 ± 3.88
Height (cm)	Patient's height	152.67 ± 7.09	151.75 ± 5.09
Weight (kg)	Patient's weight	63.61 ± 14.03	65.21 ± 10.01
BMI (mm)	Body mass index	27.28 ± 5.70	28.31 ± 4.02
BMD (g/cm^2^)	Total Bone Mineral Density	0.70 ± 0.13	0.8 ± 0.1

**Table 2:** Geometrical attributes.

	Geometrical attributes		
Attribute	Description	Fractured (mean ± SD)	Control (mean ± SD)
NW (mm)	Neck width	29.29 ± 2.02	29.68 ± 2.32
HAL (mm)	Hip axis length	89.74 ± 6.31	88.98 ± 5.48
NSA (^o^)	Neck-shaft axis angle	126.48 ± 6.11	124.21 ± 6.24
SAL (mm)	Shaft axis length	83.16 ± 5.34	85.79 ± 5.19
ITW (mm)	Intertrochanteric width	50.29 ± 3.12	50.15 ± 3.32
STW(mm)	Subtrochanteric width	27.65 ± 2.17	26.44 ± 1.52
FA (mm^2^)	Proximal femur area	4580.09 ± 490.35	4574.10 ± 372.61

**Table 3:** Fall-related attributes.

	Fall-related attributes		
Attribute	Description	Fractured (mean ± SD)	Control (mean ± SD)
STH (mm)	Soft tissue thickness	30.43 ± 13.43	32.85 ± 9.42
FPK (N)	Peak impact force	5206.08 ± 641.10	5284.01 ± 455.86
FAT (N)	Attenuation force	2160.27 ± 947.06	2332.19 ± 668.80
FP (N)	Impact force	3045.81 ± 518.10	2951.82 ± 371.04
HP (MPa)	Hip pressure	6.74 ± 1.14	6.46 ± 0.87

**Table 4:** Attributes related to the bone tissue.

	Bone tissue related attributes		
Attribute	Description	Fractured (mean ± SD)	Control (mean ± SD)
TB (%)	Percentage of trabecular bone	86.94 ± 9.04	82.10 ± 8.92
TBE (GPa)	Average Young's modulus of trabecular bone	3.59 ± 0.53	3.85 ± 0.39
CT (%)	Percentage of cortical bone	13.06 ± 9.04	17.90 ± 8.92
CTE (GPa)	Average Young's modulus of cortical bone	10.89 ± 1.96	11.57 ± 1.00

**Table 5:** Attributes obtained from the FE analysis of the side fall.

	FE analysis attributes		
Attribute	Description	Fractured	Control
N = neck; T = trochanter		(mean ± SD)	(mean ± SD)
LSR	Load-to-strength-ratio	0.98 ± 0.65	0.63 ± 0.28
FS (N)	Femoral strength	4421.34 ± 2553.70	5285.70 ± 1718.72
S1_N (MPa)	Maximum principal stress	1.49 ± 0.40	1.46 ± 0.36
S3_N (MPa)	Minimum principal stress	−3.88 ± 0.77	−3.81 ± 0.68
E1_N (*μ*strain)	Maximum principal strain	1042.10 ± 430.64	816.49 ± 180.71
E3_N (*μ*strain)	Minimum principal strain	−2250.30 ± 1016.03	−1689.79 ± 400.75
MPStress_N (MPa)	Major principal stress	5.15 ± 1.07	5.12 ± 0.94
MPStrain_N (*μ*strain)	Major principal strain	2353.53 ± 1034.01	1784.85 ± 414.42
SDE_N (J/m^3^)	Strain energy density	7473.06 ± 4113.33	5669.81 ± 1903.91
S1_T (MPa)	Maximum principal stress	0.40 ± 0.13	0.38 ± 0.11
S3_T (MPa)	Minimum principal stress	−2.94 ± 0.55	−2.84 ± 0.49
E1_T (*μ*strain)	Maximum principal strain	689.95 ± 363.99	499.23 ± 124
E3_T (*μ*strain)	Minimum principal strain	−1457.57 ± 875.67	−1105.74 ± 273.43
MPStress_T (MPa)	Major principal stress	3.24 ± 0.59	3.12 ± 0.52
MPStrain_T (*μ*strain)	Major principal strain	1571.41 ± 883.43	1122.79 ± 276.95
SDE_T (J/m^3^)	Strain energy density	3536.94 ± 2194.64	2540.23 ± 896.58
FRI_N (*μ*strain)	Fracture risk index	0.32 ± 0.14	0.24 ± 0.06
FRI_T (*μ*strain)	Fracture risk index	0.21 ± 0.12	0.15 ± 0.04

**Table 6:** Percentage of variance included in the 39 components of the PCA.

PC1	PC2	PC3	PC4	PC5	PC6	PC7-39
91.88%	5.28%	2.16%	0.38%	0.26%	0.04%	0%

**Table 7:** Variables whose correlation is higher than 0.9 and was not included by PCA are shown in the columns. The rows show variables that are highly correlated with the column attributes, coded by the check sign.

	HP	S3_N	StressN	StrainN	E1_T	E3_T	StressT	StrainT	FRI_N	FRI_T	Final
STW		✓									✓
HP		✓	✓				✓				✓
TBE		✓									✓
CTE		✓									✓
S3_N	✓		✓								✓
E1_N				✓					✓		✓
E3_N				✓					✓		✓
StressN	✓	✓					✓				✓
StrainN								✓	✓		✓
SED_N				✓				✓	✓		✓
S3_T	✓		✓				✓				✓
E1_T						✓				✓	✓
E3_T					✓					✓	✓
StressT	✓		✓								✓
StrainT					✓	✓				✓	✓
SED_T					✓	✓		✓		✓	✓
FRI_N				✓							✓
FRI_T					✓	✓		✓			✓

**Table 8:** Attributes directly included and those included because of their high correlation (≥0.9).

Directly included	Correlation ≥ 0.9	
BMI	Weight	S3_T
FPK	STH	E1_T
FP	TBE	E3_T
HP	CTE	MPStress_T
TB	E1_N	MPStrain_T
S3_N	E3_N	SED_T
FRI_N	MPStress_N	FAT
FRI_T	MPStrain_N	STH
	SED_N	CT

**Table 9:** Results for Logistic Regression with the selected 8 features.

8 features	Mean	St. deviation	Best
Sensitivity	68.22%	12.61%	94.44%
Specificity	72.69%	12.77%	84.61%
Accuracy	70.10%	8.92%	90.32%

**Table 10:** Results for Logistic Regression with 12 features.

12 features	Mean	St. deviation	Best
Sensitivity	70.33%	12.31%	100.00%
Specificity	71.46%	13.62%	84.61%
Accuracy	70.81%	10.15%	93.54%

**Table 11:** Results of SVM with a linear kernel.

Linear	Mean	St. deviation	Best
Sensitivity (8 features)	61.22%	10.20%	83.33%
Specificity (8 features)	76.69%	10.85%	92.30%
Accuracy (8 features)	67.71%	8.81%	87.10%
Sensitivity (12 features)	68.44%	9.76%	88.89%
Specificity (12 features)	75.62%	13.35%	92.30%
Accuracy (12 features)	71.45%	9.17%	90.32%

**Table 12:** Results of SVM with a linear kernel and posterior probability regions.

Linear + PPR	Mean	St. deviation	Best
Sensitivity (8 features)	63.94%	9.75%	88.89%
Specificity (8 features)	75.08%	12.28%	100.00%
Accuracy (8 features)	68.61%	9.05%	93.54%
Sensitivity (12 features)	68.17%	9.63%	88.89%
Specificity (12 features)	77.23%	12.17%	92.31%
Accuracy (12 features)	71.97%	8.71%	90.32%

**Table 13:** Results of SVM with a sigmoid kernel.

Sigmoid	Mean	St. deviation	Best
Sensitivity (8 features)	56.33%	12.61%	77.78%
Specificity (8 features)	60.62%	14.35%	84.61%
Accuracy (8 features)	58.13%	9.17%	80.65%
Sensitivity (12 features)	56.50%	12.41%	66.67%
Specificity (12 features)	60.77%	14.36%	100.00%
Accuracy (12 features)	58.29%	9.16%	80.65%

**Table 14:** Results of SVM with a sigmoid kernel and posterior probability regions.

Sigmoid + PPR	Mean	St. deviation	Best
Sensitivity (8 features)	55.39%	12.37%	77.78%
Specificity (8 features)	59.23%	14.40%	84.62%
Accuracy (8 features)	57.00%	10.09%	80.65%
Sensitivity (12 features)	55.94%	11.23%	83.33%
Specificity (12 features)	58.38%	15.66%	69.23%
Accuracy (12 features)	56.97%	8.67%	77.41%

**Table 15:** Results of SVM with a Bayesian kernel and posterior probability regions.

Bayesian + PPR	Mean	St. deviation	Best
Sensitivity (8 features)	56.67%	2.48%	55.56%
Specificity (8 features)	80.00%	6.88%	84.62%
Accuracy (8 features)	66.45%	2.89%	67.74%
Sensitivity (12 features)	71.11%	3.51%	77.78%
Specificity (12 features)	80.77%	8.31%	92.31%
Accuracy (12 features)	75.16%	4.57%	83.87%

**Table 16:** Results of SVM with a Gaussian kernel.

Gaussian	Mean	St. deviation	Best
Sensitivity (8 features)	82.56%	9.24%	88.89%
Specificity (8 features)	66.31%	14.90%	100.00%
Accuracy (8 features)	75.74%	8.23%	93.54%
Sensitivity (12 features)	96.22%	5.05%	100.00%
Specificity (12 features)	58.08%	15.09%	76.92%
Accuracy (12 features)	80.23%	6.96%	90.32%

**Table 17:** Results of SVM with a Gaussian kernel and posterior probability regions.

Gaussian + PPR	Mean	St. deviation	Best
Sensitivity (8 features)	86.22%	9.39%	100.00%
Specificity (8 features)	63.38%	15.35%	100.00%
Accuracy (8 features)	76.65%	8.97%	100.00%
Sensitivity (12 features)	93.67%	5.91%	100.00%
Specificity (12 features)	62.92%	16.56%	92.31%
Accuracy (12 features)	80.77%	7.57%	96.77%

**Table 18:** Results of Decision Trees.

Decision Tree	Mean	St. deviation	Best
Sensitivity (8 features)	59.22%	13.91%	88.89%
Specificity (8 features)	73.08%	12.46%	84.62%
Accuracy (8 features)	65.03%	8.85%	87.10%
Sensitivity (12 features)	59.67%	15.46%	99.44%
Specificity (12 features)	74.46%	18.09%	92.31%
Accuracy (12 features)	65.87%	11.66%	93.55%

**Table 19:** Results of Random Forest.

	8 features	12 features
Sensitivity	79.50	83.33%
Specificity	87.75	92.31%
Accuracy	82.66	87.10%

## Data Availability

The data used to support the findings of this study are restricted by ASCIRES company in order to protect patient privacy. Data are available from María José Rupérez for researchers who meet the criteria for access to confidential data.
